# HDAC6 inhibitor TST strengthens the antiproliferative effects of PI3K/mTOR inhibitor BEZ235 in breast cancer cells via suppressing RTK activation

This article has been retracted.

**DOI:** 10.1038/s41419-018-0931-0

**Published:** 2018-09-11

**Authors:** Shixiu Sun, Yujie Zhang, Jianchao Zheng, Biao Duan, Jie Cui, Yan Chen, Wenjie Deng, Bixing Ye, Lei Liu, Yongchang Chen, Jun Du, Luo Gu

**Affiliations:** 1 Department of Physiology, Nanjing Medical University, Nanjing, Jiangsu 211166 China; 2 Key Laboratory of Cardiovascular & Cerebrovascular Medicine, School of Pharmacy, Nanjing Medical University, Nanjing, Jiangsu 211166 China; 3 Jiangsu Key Lab of Cancer Biomarkers, Prevention and Treatment, Collaborative Innovation Center For Cancer Personalized Medicine, Nanjing Medical University, Nanjing, Jiangsu 211166 China; 4 BGI Education Center, University of Chinese Academy of Sciences, Shenzhen, Guangdong 518083 China; 5 Department of Physiology, Xuzhou Medical University, Xuzhou, Jiangsu 221004 China; 6 Department of Biochemistry and Molecular Biology, Nanjing Medical University, Nanjing, Jiangsu 211166 China; 7 Department of Gastroenterology, The First Affiliated Hospital of Nanjing Medical University, Nanjing, Jiangsu 210029 China; 8 Department of Physiology, School of Medicine, Jiangsu University, Zhenjiang, Jiangsu 212013 China

## Abstract

NVP-BEZ235 (BEZ235), an available dual PI3K/mTOR inhibitor, showed antitumor effect and provided a therapy strategy in carcinomas. However, the acquired upregulation of multiple receptor tyrosine kinases (RTKs) by NVP-BEZ235 in tumors limits its clinical efficacy. HDAC6, a class II histone deacetylase, is associated with expressions of multiple RTKs. The aim of this study was to detect whether co-treatment with HDAC6 inhibitor Tubastatin A (TST) would enhance the anticancer effects of BEZ235 in breast cancer cells. In this study, we described that treatment of breast cancer cell lines (T47D, BT474, and MDA-MB-468) with BEZ235 significantly triggered PI3K/mTOR signaling inactivation and increased multiple RTK expression, including EGFR, HER2, HER3, IGF-1 receptor, insulin receptor, and their phosphorylation levels. The adding of TST destabilized these RTKs in those breast cancer cells. Co-treatment with BEZ235 and TST reduced cell proliferative rate by strengthening Akt inactivation. In addition, the combination of these two drugs also cooperatively arrested cell cycle and DNA synthesis. In conclusion, the co-treatment with PI3K/mTOR inhibitor BEZ235 and HDAC6 inhibitor TST displayed additive antiproliferative effects on breast cancer cells through inactivating RTKs and established a rationable combination therapy to treat breast cancer.

## Introduction

Breast cancer, the most frequently diagnosed malignancy, is the second leading reason of death among women worldwide^1^. Although the early diagnosis of breast cancer has made great progress, about 30% of these patients were relapsed eventually^2^. Traditional breast cancer therapy such as chemotherapy, radiotherapy, and endocrine therapy has strong side effect. Therefore, new therapeutic strategies are attracting more and more attention to improve therapeutic efficacy.

Molecularly targeted therapy, which aims at mutations or dysregulated pathways leading to oncogenesis, is a popular modality of pharmacotherapy for cancer in recent years^3^. PI3K/AKT/mTOR signaling plays an important role in responding to various extracellular growth factors and regulates different cellular processes, including proliferation, survival, differentiation, and angiogenesis. Since this signaling is frequently dysregulated in cancer^4^, several drugs targeting PI3K, AKT, or mTOR have been used to treat patients with breast cancer generally. However, the clinical efficacy of those inhibitors was limited because of the upregulation of receptor tyrosine kinases (RTKs) induced by themselves^5–8^. Therefore, whether co-treatment with other drugs targeting other carcinogenic sites to abrogate the upregulation of RTKs is a question deserving further research in breast cancer therapy.

BEZ235, a class I dual inhibitor of PI3K/mTOR, has great potential as an antitumor drug, which undergoes evaluation in phase I/II clinical trials currently^9–11^. Recent studies indicated BEZ235 inhibited PI3K signaling transiently and its therapeutic effects in ovarian cancer and breast cancer were not efficient^12^. Studies have shown that combinatorial targeted therapy may be more effective compared with single agent in treating cancer by blocking by-pass mechanisms or inducing synthetic lethality^13^. Recent clinical studies showed that BEZ235 exhibits synergistic antitumor effects with other chemotherapeutic agents in several different types of cancers, including prostate cancer, lung cancer, neuroblastoma, etc^14^. HDAC6, a class II histone deacetylase, is overexpressed in breast cancer cells^15^. HDAC6 acts as a deacetylase for HSP90, α-tubulin, and cortactin. Targeted inhibition of HDAC6 has been shown to induce acetylation of HSP90 and disruption of its chaperone function^16^. Recent studies have reported that HSP90 is positively correlated with RTK expression^17–19^. Tubastatin A (TST) is a selective inhibitor of HDAC6. Thus, we hypothesized that co-treatment of BEZ235 and TST would exert the synergistic therapeutic effect on breast cancer cells.

In this study, we found that BEZ235 induced upregulation of RTKs in breast cancer cells, including total protein of epidermal growth factor receptor (EGFR), HER2, HER3, insulin receptor, and insulin-like growth factor-1 (IGF-1) receptor, and their phosphorylation levels. Co-treatment with TST abrogated the upregulation of RTKs induced by BEZ235. The combination of these two drugs also cooperatively arrested cell cycle in G1/S phase and inhibited breast cancer cell proliferation. Our study established a rationable combination therapy with BEZ235 and TST, which may have a potential clinical perspective in breast cancer treatments.

## Results

### BEZ235 treatment suppressed PI3K/AKT/mTOR signaling and cell viability of breast cancer cells

Three breast cancer cell lines (T47D, BT474, and MDA-MB-468) were chosen to detect appropriate drug concentration of BEZ235. The genotype of T47D is ER^+^, PR^+^, and PI3K-mutated; the genotype of BT474 is HER2^+^ and PI3K-mutated, while the genotype of MDA-MB-468 is ER/PR/HER2-negative. The breast cancer cells were treated with different doses of BEZ235 for 24 h. Then the activations of p70S6K and AKT, the main downstream proteins of PI3K, were detected. The concentration of BEZ235 used here was in good consistency with previous studies^20^. The results showed that expression of p-p70S6K and p-AKT (S473) decreased with increasing concentration of BEZ235, but p-AKT (T308) expression increased in T47D and MDA-MB-468 cells (Fig. 1a and Figure S1a). Similar alterations were found in BT474 cells despite the suppression of p-p70S6K and p-AKT was achieved by lower concentration of BEZ235 (Fig. 1b). As shown in Fig. 1c, d and Figure S1b, BT474 inhibited breast cancer cell proliferation in a concentration-dependent manner. According to the above results, 100 nM BEZ235 was chosen to treat T47D and BT474 cells, 200 nM was chosen for MDA-MB-468 in the following experiments.

**Fig. 1:** BEZ235 suppressed PI3K/AKT/mTOR signaling and cell viability. **a** T47D and **b** BT474 cells were treated with DMSO or different concentrations of BEZ235 for 24 h. Whole-cell lysates were prepared, and western blot analyses were performed to detect p-p70S6K, p70S6K, AKT, p-AKT (S473), and p-AKT (T308). **c** T47D and **d** BT474 cells were exposed to increasing doses of BEZ235 for 24 h. Cell viability was evaluated by MTT assay. **P *<* 0.01 versus control group. Data shown are mean ± SEM of at least three independent experiments

### Expressions of multiple RTKs were induced by BEZ235

It is previously revealed that inhibition of PI3K, AKT, or mTOR is involved in the upregulation of multiple RTKs, including ERBB family, insulin receptor, IGF-1 receptor, and so on^6,7,21–23^. Among these detected RTKs, EGFR, HER2, and HER3 were widely studied and targeted in breast cancer cells while the therapeutic impact and prognostic of HER4 expression remain unclear^23,24^. Insulin receptor and IGF-1 receptor were also closely related to drug resistance and their expression was detected as well. BEZ235 is a class I dual inhibitor of PI3K/mTOR. To elucidate the effect of BEZ235 on RTKs, T47D and BT474 cells were treated with BEZ235 for 48 h and expressions of RTKs were detected. As shown in Fig. 2a, b and Figure S2a, total protein levels of these RTKs increased and their phosphorylation levels also had a rising trend after BEZ235 treatment in the three breast cancer cell lines. Consistently, the mRNA levels of EGFR, HER2, HER3, HER4, insulin receptor, IGF-1 receptor, insulin receptor substrate-1 (IRS-1), MET, platelet-derived growth factor (PDGF) receptor A, PDGF receptor B, vascular endothelial growth factor (VEGF) receptor 2, RYK, fibroblast growth factor receptor (FGFR), and ROR2 were increased under the same treatment (Fig. 2c, d and Figure S2c).

**Fig. 2:** BEZ235-induced expression and phosphorylation of multiple RTKs. **a** T47D and **b** BT474 cells were treated with BEZ235 (100 nM) for the indicated times. The expression of RTKs and their phosphorylation levels were detected by western blot analyses. **c**, **d** Some RTKs’ mRNA levels in T47D and BT474 cells were detected by qPCR. **e** T47D and **f** BT474 cells were treated with BEZ235 (100 nM) for 36 h and the cellular lysates were applied to p-RTK arrays. Spots are in duplicate and each pair corresponds to a specific p-RTK. **g** T47D and **h** BT474 cells were treated with BEZ235 (100 nM) for 48 h. Downstream signals of RTKs were also detected. *P < 0.05; **P *<* 0.01 versus control group. Data shown are mean ± SEM of at least three independent experiments

We also treated T47D and BT474 cells with BEZ235 and the cellular lysates were applied to phospho-RTK array, which reflects phosphorylation status of 49 RTKs. Consistent with Fig. 2a, the results of Fig. 2e showed that the expressions of P-HER2, P-HER3, and P-HER4 were obviously increased after BEZ235 treatment in T47D cells. The results also showed the increase of P-ROR2 and P-RYK. Since these two RTKs are associated with Wnt signaling, it deserves further study to explore whether PI3K/AKT signaling and Wnt signaling have crosstalk in BEZ235 treatment. As shown in Fig. 2f, phosphorylation of ERBB family (EGFR, HER2, HER3, and HER4), FGFR, insulin receptor, IGF-1 receptor, ROR2, and RYK was increased after BEZ235 treatment in BT474. The quantification of the signals and their normalized expression were shown in Figure S10. Together, these results suggested that BEZ235 treatment could not only inhibit PI3K/mTOR pathway but also induce the expression and activation of multiple RTKs.

To make it clear whether RTK expression could lead to an reactivation of PI3K/mTOR signaling after BEZ235 treatment, p-AKT and p-p70S6K status were detected for 48 h (Fig. 2g, h and Figure S2b). The results showed that p-p70S6K was gradually decreased and persistent to be inhibited; p-AKT (S473) and p-AKT (T308) were inhibited to a low level in first 8 h and subsequently increased gradually. These results indicated that treatment of BEZ235 led to reactivation of PI3K/AKT signaling, which would impair its clinical efficacy.

### Expressions of multiple RTKs were suppressed by HDAC6 inhibitor TST

HDAC6 was a unique cytoplasmic deacetylase, targeting tubulin, HSP90, and cortactin^25^, and directly or indirectly correlated with multiple RTKs^26–31^. We treated T47D, BT474, and MDA-MB-468 cells with the selective HDAC6 inhibitor TST. By western blotting assay, we found that acetylation of α-tubulin was upregulated by TST dose-dependently (Fig. 3a, b and Figure S3a), which indicated TST affected enzymatic activity of HDAC6. The results of cell viability showed that inhibitory rate reached 15% at 10–15 μM TST (Fig. 3c, d and Figure S3b). Subsequently, 10 μM TST was used to treat T47D and 15 μM TST was used to treat BT474 and MDA-MB-468 cells for the next experiments. The results showed that after 48 h incubation, levels of total EGFR, HER2, HER3, insulin receptor, and IGF-1 receptor, and levels of P-EGFR, P-HER2, and P-HER3 were downregulated differently (Fig. 3e, f and Figure S3c). To further confirm the effect of TST on PI3K/AKT signaling, p-p70S6K, p-AKT (S473), p-AKT (T308), and acetylated-α-tubulin were detected by western blotting. As shown in Fig. 3g, h and Figure S3d, the levels of p-p70S6K, p-AKT (S473), and p-AKT (T308) were decreased gradually while acetylation of α-tubulin was persistently at a high level. Collectively, the present results indicated that TST may downregulate multiple RTKs and suppress PI3K/AKT/mTOR signaling.

**Fig. 3:** HDAC6 inhibitor TST repressed RTK expression. **a** T47D and **b** BT474 cells were treated with different concentrations of TST for 24 h. Western blot analyses were performed to detect α-tubulin and its acetylation level. **c** T47D and **d** BT474 cells were exposed to increasing doses of TST for 24 h. Cell viability was evaluated by MTT assay. **e** T47D cells were treated with 10 μM TST and **f** BT474 cells were treated with 15 μM TST for indicated times. Indicated proteins were detected by western blot. **g**, **h** PI3K/AKT/mTOR signaling and acetylation of α-tubulin were detected under the same treatment in T47D and BT474 cells. *P < 0.05, **P < 0.01, and ***P < 0.001 versus control group. Data shown are mean ± SEM of at least three independent experiments

### TST abrogated survival pathways induced by BEZ235

Recent study showed the clinical efficiency of BEZ235 on breast cancer was limited^12^. Whether this restriction was due to RTKs’ upregulation, and the combination of BEZ235 and RTKs inhibitors would be more effective? Next, we investigated whether TST could abrogate BEZ235-induced upregulation of RTKs. As expected, TST treatment alone downregulated most tested RTKs’ protein levels in these three breast cancer cell lines while BEZ235 upregulated the expression of these proteins. Accordingly, upregulation of EGFR, HER2, HER3, insulin receptor, and IGF-1 receptor induced by BEZ235 was suppressed by TST co-treatment (Fig. 4a, b and Figure S4a).

**Fig. 4:** TST suppressed survival pathways induced by BEZ235. **a** T47D and **b** BT474 cells were stimulated with BEZ235 and TST for 36 h. Total protein and their phosphorylation levels of RTKs were detected by western blot. **c**, **d** To further demonstrate the downstream signal changes, p-S6K, p-AKT, and acetylated-α-tubulin were also detected in both cell lines. **e** T47D and **f** BT474 cells were treated with BEZ235 and TST for 36 h, cellular lysates were applied to p-RTK arrays

As AKT and p70S6K are downstream effectors of multiple RTKs, we next evaluated the effects of combination of BEZ235 and TST on these proteins (Fig. 4c, d and Figure S4b). We found that p-AKT (S473) and p-p70S6K were suppressed by BEZ235 and TST respectively and co-treatment with these two drugs enhanced these effects. Compared with BEZ235, p-AKT (T308) was also inhibited by co-treatment of BEZ235 and TST.

To further determine the effects of the two drugs, phospho-RTK arrays were applied to T47D and BT474 cells, which were treated with BEZ235 and TST. As shown in Fig. 4e, f, in T47D cells, co-treatment of BEZ235 and TST decreased the phosphorylation of EGFR, HER2, HER3, HER4, ROR2, and RYK compared with BEZ235 group. In BT474 cells, combination treatment led to downregulation of phosphorylation of ERBB family, insulin receptor, IGF-1 receptor, ROR2, and RYK in contrast with BEZ235 alone. The quantification of the signals and their normalized expression were shown in Figure S10. These results implied that combined treatment of the two drugs may be more effective on treating breast cancer.

### Additive effect of BEZ235 and TST on inhibiting cell proliferation

To determine the effect of BEZ235 and TST on cell proliferation, several functional studies were performed. The results of MTT assays showed co-treatment with BEZ235 and TST could significantly inhibited breast cancer cell viability (Fig. 5a, b and Figure S5a). According to *Q* value method of Zhengjun jin^32^ (*Q* value > 1.15 was synergistic; 0.85–1.15 was additive; <0.85 was antagonistic), combination of BEZ235 and TST had addictive effect.

**Fig. 5:** Co-treatment with BEZ235 and TST synergistically inhibited breast cancer cell proliferation. **a** T47D and **b** BT474 cells were treated with BEZ235 and TST for indicated times. Viable cells were measured by MTT assays. **c** T47D and **d** BT474 cells were treated with BEZ235 and TST for 24 h. The cells were then cultured for 2 weeks and the colonies were photographed. **P < 0.01, ***P < 0.001 versus control group. Data shown are mean ± SEM of at least three independent experiments

The results of colony formation assays showed that co-treatment with BEZ235 and TST significantly inhibited colony formation of T47D, BT474, and MDA-MB-468 cells (Fig. 5c, d and Figure S5b).

Proapoptotic effect in the combination therapy was also presented. By staining cells with a combination of fluorescein annexin V-fluorescein isothiocyanate (FITC) and propidium iodide (PI), it is possible to distinguish and quantitatively analyze non-apoptotic cells (annexin V-FITC-negative/PI-negative), early apoptotic cells (annexin V-FITC-positive/PI-negative), late apoptotic/necrotic cells (annexin V-FITC-positive/PI-positive), and dead cells (annexin V-FITC-negative/PI-positive) through flow cytometry. In Figure S8, we found no distinct proapoptotic effect in the combination therapy.

These results highlighted the inhibitory effects of BEZ235 and TST on breast cancer cell proliferation in vitro.

### BEZ235 and TST synergistically induced cell cycle arrest and inhibited DNA synthesis

We further examined whether this antiproliferation effect of BEZ235 and TST was due to cell cycle arrest. The breast cancer cells of three genotypes were co-treated with BEZ235 and TST for 36 h and the cycle phase distribution was measured. As shown in Fig. 6a, b and Figure S6a, BEZ235 or TST induced G1 phase arrest and their co-treatment greatly enhanced cell accumulation in G1 phase, which accompanied by a reduction in S phase. The expression of the main cell cycle relative proteins was also analyzed by western blotting (Fig. 6e, f). Co-treatment with BEZ235 and TST decreased the expression of cyclin D1, cyclin E1, CDK2, CDK4, and CDK6.

**Fig. 6:** BEZ235 and TST displayed synergistic effect on cell cycle arrest. **a** T47D and **b** BT474 cells were treated with BEZ235 and TST for 36 h. Cells were then trypsinized, washed, and re-suspended in 1× binding buffer. Cell cycle distribution was studied by using flow cytometry following PI staining. **c**, **d** Data of cell cycle distribution were calculated. **e** T47D and **f** BT474 cells were treated with BEZ235 and TST for 36 h. Cell cycle-related proteins were detected by western blotting

To study the influence of BEZ235 and TST on DNA synthesis, we conducted 5-ethynyl-2′-deoxyuridine (EdU) assays. EdU is a thymidine analog with a few alkyne groups that are rare in natural compounds and can substitute for thymine (T) during DNA replication. As shown in Fig. 7a, b and Figure S7, these results indicated that co-treatment with BEZ235 and TST significantly inhibited DNA synthesis of breast cancer cells. In conclusion, the co-treatment with these two drugs demonstrated additive effect against cell proliferation in breast cancer cells and established a rational combination approach in the breast cancer therapy.

**Fig. 7:** BEZ235 and TST displayed synergistic effect on DNA synthesis inhibition. **a** T47D and **b** BT474 cells were seeded in 96-well plate and treated with TST plus BEZ235 for 36 h. Then, EdU was added to each well for 2 h. Images were taken by using fluorescence microscopy. **c**, **d** EdU-positive cell was calculated with (EdU add-in cells/Hoechst-stained cells) × 100%. ***P < 0.001. Data shown are mean ± SEM of at least three independent experiments, scale bar: 30 μm

## Discussion

The PI3K/AKT/mTOR pathway is often dysregulated in cancer cells^33^. Since targeting PI3K, AKT, mTORC1, or mTORC2 sites are reported to induce feedback activation of some survival signalings^6,8,34^, cancer cells can escape from single drug treatment, which only targeting PI3K/AKT. Thus, inhibiting these aberrant activation proteins and rationally designing combinations therapies will pave ways for breast cancer treatment^23^. In this study, we found that TST exerted additive effects with BEZ235 in inhibition of breast cancer cell proliferation. Our further study revealed that inactivations of RTKs and PI3K/AKT signaling were involved in the anti-breast cancer effects.

Consistent with the findings of Muranen et al.^12^, we noticed here that in breast cancer cells, inhibition of PI3K/mTOR signaling by BEZ235 induced upregulation of total protein and phosphorylation levels of EGFR, HER2, HER3, insulin receptor, and IGF-1 receptor. Upregulation of RTKs is reported to increase cancer cell resistance to inhibitor of PI3K/AKT/mTOR pathway^6,8^. Since the inhibition of mTORC1 and p70S6K by BEZ235 may activate FOXO, and then accelerate those receptors’ transcription and expression^6^, we speculated that in breast cancer cells, the upregulation of RTKs induced by BEZ235 may also depend on FOXO activity. Based on the diversity and complexity of these increased oncogenic RTKs, it is unrealistic to suppress those RTKs with multiple drugs.

HDAC6 has unique cyto-protective function that depends on its ability to prevent protein aggregation^35^. It has been reported that HDAC6 is associated with several carcinogenic RTKs, including EGFR, HER2, VEGFR, and PDGFR via tubulin, HSP90, and some ubiquitin-related proteins^27,36^. Thus, HDAC6 inhibition might cause changes of RTKs. In our studies, we found that HDAC6 inhibitor TST decreased the expressions of EGFR, HER2, HER3, insulin receptor, and IGF-1 receptor, and there were no significant changes in their mRNA levels (Figure S9). It was reported that HDAC6 prevented RTKs’ degradation by inhibiting RTK transport to late endosome^37^. Therefore, it is proposed that TST induces downregulation of RTKs through enhancing their degradation. TST treatment also caused time-dependent inactivation of AKT and p70S6K. In addition to our work, other studies also showed that inhibition of HDAC6 contributed to tumor inhibition by activating PTEN^38,39^, implying that targeting HDAC6 may achieve efficacy in cancer therapy.

Although it is well studied on PI3K/AKT/mTOR pathway and their inhibitors, no studies have described the resistance mechanisms of BEZ235 and evaluated the efficacy of combination therapy, including BEZ235 in breast cancer. Combination therapy is an important strategy for improving therapeutic efficacy for cancer, it may avoid drug resistance and dealing with the complexity of signaling pathway network^23^. Based on the reaction of co-treatment with BEZ235 and TST on RTKs, and the enhanced inhibition of cell proliferation, cell cycle, and DNA synthesis, it would be a new strategy to use both BEZ235 and TST on breast cancer therapy.

## Materials and methods

### Cell lines and cell culture

Human breast cancer cell lines (T47D, BT474, and MDA-MB-468) were obtained from the Cell Biology Institute of Chinese Academy of Sciences (Shanghai, China). T47D and MDA-MB-468 cells were cultured in Dulbecco’s modified Eagle’s medium (high glucose) (Biological Industries, USA). BT474 cells were cultured in RPMI 1640 medium (Biological Industries, USA), supplemented with 10% (v/v) fetal bovine serum (Gibco, USA) and maintained at 37 °C with 5% CO_2_^40,41^.

### Reagents

BEZ235 was obtained from ApexBio Technology (USA) and TST was purchased from Selleck chemicals (USA).

### Western blotting

Extraction and concentration determination of sample protein were performed as previously described^41^. Equal amount of protein from different samples was loaded on SDS polyacrylamide gels, then were transferred to nitrocellulose membrane. After blocking with Tris-buffered saline (TBS) containing 5% fat-free milk, the blots were incubated with primary antibodies overnight at 4 ℃ and horseradish peroxidase (HRP)-conjugated secondary antibodies (Santa Cruz, CA, USA) for 1 h at room temperature. Rabbit antibodies against p-AKT (473), p-AKT (308), AKT, and p70S6K, and mouse antibody against p-p70S6K were purchased from Cell Signaling Technology (Danvers, MA, USA). Antibodies against EGFR, HER2, HER3, acetyl-α-tubulin, cyclin D, cyclin E, CDK2, CDK4, CDK6, and actin were purchased from Santa Cruz (USA). Antibodies against p-HER2 (Tyr1248) and p-HER3 (Tyr1289) were purchased from Affinity (China). Antibodies against p-EGFR (Tyr 1069) and α-tubulin were purchased from Abscience (China). Subsequently, the blots were washed with TBST for three times, incubated with ECL reagent (Millipore, USA), and visualized by ChemiDoc XRS+ gel imaging system (Bio-Rad, USA). Image gray value analysis was performed by ImageJ (NIH, USA) and the intensities of actin were used as a control for all other bands^40^.

### RTK arrays

The human p-RTK array kit (R&D System, Inc.) was used to detect the level of RTK phosphorylation. Cells were treated with dimethyl sulfoxide (DMSO) or drugs for 36 h and then lysed with lysis buffer, 300 μg proteins were processed according to the manufacturer’s protocols. Briefly, these arrays were incubated with cell lysates overnight with shaking at 4 ℃ and then washed with washing buffer for three times. Arrays binding with target protein were then incubated with anti-p-tyrosine-HRP detection antibody with rocking for 2 h at room temperature. The arrays were washed and incubated chemiluminescent reagent, and finally exposed by ChemiDoc XRS+ gel imaging system (Bio-Rad, USA).

### Quantitative reverse transcription PCR

Quantitative reverse transcription PCR (qPCR) was performed as previously described^41^. Total RNAs from cells were extracted with TRIzol reagent (Invitrogen, Pleasanton, CA, USA). Equal amounts of RNA (5 μg) of each sample were used to synthesize cDNA using HiScriptQ RT SuperMix (Vazyme, Nanjing, China). qPCR was performed on the ABI StepOne™ Real-Time PCR System (Applied Biosystems, Foster City, CA, USA) using AceQ qPCR SYBR Green Master Mix assay (Vazyme, Nanjing, China) and analyzed using StepOne Software v2.1 (Applied Biosystems). Gene expression levels were calculated by relative quantification (2^−ΔΔCT^). Primers used for qPCR amplification are available in Table 1.

**Table1:** Primer sequence

Gene	Forward primer (5′ → 3′)	Reverse primer (5′ → 3′)
*EGFR*	GGGCTCTGGAGGAAAAGAAA	AAATTCCCAAGGACCACCTC
*HER2*	CACAGAGATCTTGAAAGGAGGG	TACACATCGGAGAACAGGGG
*HER3*	GCAGTGGATTCGAGAAGTGAC	CGTGGCTGGAGTTGGTGTTAT
*HER4*	ACAGGACTTTGGGTCTGGGT	CAAGGCTCGGTACTGCTGTT
*Insulin R*	CAACGAGGAGTGTGGAGACA	GCCGTGTGACTTACAGATGGT
*IGF1R*	CAGAGCATGTACTGCATCCC	TCCCCCGTCGGATGTTAATG
*IRS1*	GGATTTGCTGAGGTCATTTAGG	TATGCCAGCATCAGTTTCCA
*MET*	ACTTTAAGTGAGAGCACGATGA	TTGTCCCGTGGCCATTTGAA
*PDGFRA*	TGGAAACAGAAACCGAGGTATG	GGCTGTTCCTTCAACCACCT
*PDGFRB*	AGACCCGGTATGTGTCAGA	ATCTGTAGCTGGAAGGAGAGC
*VEGFR2*	TCCATGTCTCGGGTCCATTT	GTAAAGCCCTTCTTGCTGTCC
*RYK*	ATACTGAGTCGTCTGGGTGGA	TAGTGTAGGGGTTTGTTGTGC
*ROR2*	GATTCGCAGTCGTGAACCATA	GACCCTTTAGGACCCCTTGAT
*FGFR3*	GCAGAGTGATGAGAAAACCCAATA	GCTAACACCACCGACAAGGAG
*Actin*	AGAGCTACGAGCTGCCTGAC	AGCACTGTGTTGGCGTACAG

### Flow cytometry

Cells were cultured in six-well plates, and subsequently treated with BEZ235, TST, or their combination. Cells were then trypsinized, washed, and re-suspended in 1× binding buffer. Cell cycle distribution was studied using flow cytometry following PI staining and proapoptotic effect was detected following annexin V and PI staining.

### Cell viability assay

Six thousand cells per well were seeded in 96-well plate. The cells were then incubated with indicated agents for different times, followed by the addition of 5 mg/mL MTT (Biosharp, China). After incubation for 4 h at 37°C, the supernatants were removed. A volume of 150 μL of DMSO were added, and the absorbance value (optical density) at 490 nm was measured by Bio-TEK system.

### Colony formation assay

One thousand cells were seeded in 35 mm dish and treated with indicated agents for 24 h. Subsequently, the cells were washed twice and cultured for up to 3 weeks. Colonies were visualized by crystal violet staining and counted according a defined colony size.

### EdU assay

Cells were seeded in 96-well plate and subsequently treated with indicated agents for 24 h. Then, 50 μM EdU (Cell Light EdU DNA imaging Kit, RiboBio, China) was added to each well, and the cells were cultured for an additional 2 h. Subsequently, cell immobilization, apollo staining, and DNA staining were performed according to the product introduction. Finally, images were taken and analyzed using fluorescence microscopy (ZEISS, Germany). Percentage of EdU-positive cells was calculated with (EdU add-in cells/Hoechst-stained cells) × 100%.

### Statistical analysis

Statistical analysis was performed by the Prism 6.0 software (GraphPad Software, USA). One-way analysis of variance was employed for multiple comparisons of means. The level of significance was set at *P* < 0.05, data were shown as mean ± SEM.

## Electronic supplementary material

Figure S1

Figure S2

Figure S3

Figure S4

Figure S5

Figure S6

Figure S7

Figure S8

Figure S9

Figure S10

supplementary figure legends
